The article "Stakeholder governance and sustainability in football: A bibliometric analysis" was published in 2023. Journal: Heliyon.

# Stakeholder governance and sustainability in football: A bibliometric analysis

**DOI:** 10.1016/j.heliyon.2023.e18942

**Published:** 2023-08-04

**Authors:** Juan Alejandro Hernández-Hernández, Abraham Londoño-Pineda, Jose Alejandro Cano, Rodrigo Gómez-Montoya

**Affiliations:** a University of Medellin, Carrera 87 # 30-65, 050031, Colombia; b Colombian Polytechnic Jaime Isaza Cadavid, Carrera 48 # 7-151, 050022, Colombia

**Keywords:** Stakeholder governance, Sustainability, Football, Soccer, Bibliometric analysis, Systematic review

## Abstract

This study presents a bibliometric analysis of stakeholder governance and sustainability in football. The PRISMA statement and the main techniques from the existing bibliometric analysis toolbox are applied to guide the research. The analysis includes 127 documents from Scopus and WoS, covering the period from 2007 to mid-2023, to examine the performance analysis and science mapping of the subject over time. The study's key findings highlight publication-related metrics, citation-and-publication-related metrics, co-authorship analysis, and co-word analysis. The analysis also identifies research gaps, including the need to explore barriers to stakeholder governance in football, the application of stakeholder pressure frameworks in football clubs, the examination of mimetic and normative pressures in the context of sustainability and governance in football, and the involvement of stakeholders and football institutions in collaborative efforts to enhance the effectiveness and impact of sustainability initiatives.

## 1 Introduction

In order to comply with the commitments outlined in the Paris Climate Agreement, both companies and governments are required to reduce their carbon emissions and contribute to Sustainable Development Goals (SDGs) achievement. In this regard, the sport has been recognized as an essential tool for the implementation of the SDGs [1], which is why sports authorities and government organizations must also work to make them part of the strategic direction of sports organizations [2]. However, despite these regulatory and governance influences, the sports sector lags behind the answers that integrate environmental and sustainability practices [3]. Indeed, the lack of prioritization of the natural environment is institutionalized within the sports sector [4]. Despite its significant economic and social impact, the football industry has lagged in addressing sustainability-oriented strategic directions [5]. Therefore, bibliometric analysis, such as the one presented in this paper, provide an opportunity to bridge the gap between competitiveness and sustainability requirements and explore the existing gaps in incorporating sustainability principles and practices within the football industry.

One of the questions arising around this issue is related to the factors that prevent companies from decisively incorporating sustainability practices, which is partly explained by the prevalence of the idea that managers only aim to ensure the maximization of shareholder profit [6]. In this sense, companies' business models have traditionally been oriented toward creating value primarily for their shareholders and customers [7]. A change of focus would imply defining current goals towards higher value ones such as sustainability [8], which would lead to expressing value not only in terms of monetary gains available to shareholders but in terms of expected economic, social and environmental outcomes [3]. It would also imply the incorporation of stakeholders to transform the idea of traditional value generation into shared value [9].

Regarding how relationships with different stakeholders can be managed, and how they can be directed toward sustainability objectives, governance represents a crucial lever to guide sporting events toward sustainability because it involves rules, systems, roles, and procedures that allow the achievement of objectives [10]. In this regard, governance and leadership failures have prevented football clubs from making progress in meeting their sustainability goals [11], so governance must link market stakeholders to improve the effectiveness of sustainability initiatives [12]. Therefore, stakeholder governance constitutes a convenient framework for studying sustainability management in organizations [12].

While there have been numerous research studies focusing on topics related to CSR in football [[13], [14], [15], [16], [17]], sustainability in sporting events [10,18,19], and environmental sustainability in football [16,20,21], it is worth noting that there is a scarcity of literature reviews and bibliometric studies that comprehensively explore the intersection of sustainability and stakeholder governance in football. Few studies specifically examine the combined aspects of sustainability and governance in relation to the key stakeholders in football. Instead, the existing literature tends to separately address reviews of CSR and football, sustainability and football, or governance and football. Therefore, there is a gap in the literature that calls for more comprehensive studies that integrate the concepts of sustainability and stakeholder governance within the context of football.

Based on the aforementioned, this study presents a bibliometric analysis of stakeholder governance and sustainability in football. The research aims to address the following three research questions.

1. Why is it important to investigate a topic that encompasses sustainability and stakeholder governance in football?
2. What is the current state of the art regarding the proposed topic in this review?
3. What potential future research directions can be identified?

The first question will be addressed in Section 2, which aims to provide a justification for conducting the bibliometric analysis. The second question will be answered in Sections 3, 4, which cover the methodology and results, respectively. The third question will guide the development of Section 5, focusing on discussions and future research directions. Finally, Section 6 presents the concluding remarks of this study.

## 2 Relevance of sustainability and governance in football

This section aims to highlight the significance of investigating the topic that encompasses sustainability and stakeholder governance in football. It begins by exploring the concepts of sustainability in football and governance in football, and subsequently emphasizes the importance of integrating these two concepts.

### 2.1 Football and its contribution to achieving sustainability goals

Football, known as soccer in some regions, has evolved to become the most popular sport globally, exerting a significant influence on various aspects of society. As stated by Alcaide [22], throughout the 20th century, football transcended the political sphere as leaders recognized its potential to foster nationalist sentiments, particularly during the FIFA World Cup tournaments that captured the attention of the masses. Notably, the 1938 World Cup played a pivotal role in unifying the fragmented national identity of Brazil, which was previously characterized by strong regionalism. This event served as a catalyst for the nation to think and act collectively. Furthermore, football has historically been associated with reinforcing religious identities, exemplified by the case of Celtic (of Catholic origin) and Rangers (of Protestant origin) in Scotland. Over time, these religious divisions have been mitigated through the unifying power of the sport. However, it was not until relatively recently in the 21st century that football began to be recognized as a significant economic activity [23]. The advent of mass media and advancements in information technology (ICT) during the 1980s and 1990s brought about substantial transformations in football, shifting its primary sources of revenue from ticket sales to advertising [24].

In the 21st century, the landscape of football has witnessed the emergence of new market options that have significantly impacted its business models. The introduction of broadcasting rights and substantial transfer fees paid for high-profile players has brought about new streams of income for football clubs [25]. However, this shift in the financial landscape has raised concerns regarding the potential erosion of traditional sports values and the weakening of the connection with fans [26]. The prioritization of financial objectives over sporting performance by some managers has been seen as contradicting the essence of the sport. Football is unique in the sense that fans form a deep emotional connection with their teams [27], making them a legitimate and influential stakeholder group with the power to influence the financial performance of football clubs [28].

The emotional connection and passion that football generates among fans sets it apart from many other sports [5]. Football teams must not only attract and retain supporters but also find ways to leverage these sentiments for profitability [29]. Interestingly, managing these emotions can also be beneficial in achieving sustainability objectives. Fans' deep passion for their teams can facilitate the development of environmental and sustainable awareness more effectively than if it were mandated by the government, a political party, or any other organization. Football, therefore, has the potential to serve as a catalyst for social change. It can transcend environmental behavior within stadiums and extend it into the personal lives of fans, contributing to society's overall sustainability goals [30].

Football teams and clubs have various motivations for pursuing sustainability goals, with financial and tax benefits being prominent factors. By embracing sustainability practices, they can not only achieve cost savings but also enhance their public image by positioning themselves as “Green Companies” [21]. However, it is important to acknowledge that organizations in the football industry often adopt environmental and sustainability initiatives in response to pressures from their stakeholders. These pressures can stem from functional, social, or political considerations, as highlighted by McCullough and Cunningham [4], McCullough and Pfahl [31], and McCullough et al. [32]. The work of Daddi et al. [33], Daddi et al. [10], and Todaro et al. [3] further supports this notion by providing evidence that European football clubs engage in sustainability initiatives and practices as a response to pressure from their stakeholders. These stakeholders can include fans, sponsors, local communities, regulatory bodies, and other stakeholders who advocate for sustainable practices and hold clubs accountable for their environmental impact. The influence of these stakeholders highlights the interconnectedness of sustainability, stakeholder governance, and the football industry.

The information provided suggests that sports, particularly football, hold the potential to drive the attainment of sustainability objectives. This potential arises from the deep emotional connection that fans have with the sport and the influence exerted by various stakeholders [4]. As a result, the relationship between sports and sustainability has gained recognition as an emerging area of research, although it is still in its early stages of development [5].

### 2.2 From corporate social responsibility to the concept of sustainability

The football industry has not been immune to international debates and movements surrounding the environment and sustainability. However, compared to other sectors, it has been slower in adopting sustainability principles, despite its significant social and economic importance [34]. One reason for this delay is that sustainability is not a mandatory requirement for football organizations. Consequently, many initiatives in this area are driven by cost savings, economic incentives, or the desire to enhance their reputation and the perception of fans and supporters [21]. Additionally, the pressure exerted by stakeholders has played a role in motivating football organizations to embrace sustainability practices [4].

Before delving into the concept of sustainability in football, it is important to differentiate between the concepts of corporate social responsibility (CSR) and sustainability. CSR emerged as a concept in the late 1970s and has since gained prominence in the research agenda of football [35,36]. More recently, the focus has shifted towards integrating CSR with environmental and sustainable development aspects [16]. In the business field, CSR has long been closely associated with sustainability [37], and while the two concepts are interconnected, they are not necessarily interchangeable [38]. Jager [39] argues that CSR is a more specific term compared to sustainability but acknowledges the increasing interest in the latter since the publication of the Bruntland report in 1987. Sustainability is seen as the natural progression of CSR, encompassing the needs of both the present and future generations, ensuring that current actions do not compromise the ability of future generations to meet their own needs [40].

Therefore, corporate sustainability encompasses both present and future performance of a company, with short-term efforts focused on minimizing economic, social, and environmental impacts, and long-term considerations addressing governance and the ethical and political stance of organizations [41]. The concept of sustainability is typically presented through the interaction of various dimensions, often based on three or four-pillar models that encompass economic, social, environmental, and sometimes institutional aspects [42]. The triple bottom line model, initially developed by Henriques and Richardson [43], has become a widely recognized representation of sustainability [7,21]. Therefore, in this study, the term sustainability refers to this model and its interconnected dimensions.

### 2.3 Stakeholder governance approach

According to Daddi et al. [33], stakeholder governance plays a crucial role in guiding sporting events towards sustainability by establishing standards, systems, roles, and procedures that enable organizations to achieve their objectives. Research suggests that stakeholder governance is essential for attaining sustainability goals. For instance, McLeod et al. [11] demonstrate that failures in governance and leadership have hindered football clubs from making advancements in their sustainability objectives. Similarly, Somjai et al. [12] propose that governance alone is significant, but combining it with market stakeholders can enhance the effectiveness of sustainability improvement initiatives for companies.

In addition to traditional governance models, different approaches to governance have emerged. Collaborative governance, for instance, emphasizes a cooperative and consensual perspective, replacing traditional top-down management models with new administrative forms based on negotiation and coordination among stakeholders [44]. Participatory governance is another approach where stakeholders are actively involved in the decision-making and management of organizations, thereby influencing the performance outcomes [26]. These alternative governance approaches recognize the importance of engaging multiple stakeholders and fostering inclusive processes in achieving sustainability objectives.

The analysis of governance failures in football organizations has highlighted several key issues, including deficient communication practices by managers, limited inclusion of fans in advisory or decision-making roles, and barriers to active fan participation with a bottom-up approach. Todaro et al. [3] emphasize that football involves various types of stakeholders, including football institutions such as FIFA, UEFA, CONMEBOL, government institutions at national and local levels, as well as market and stakeholders such as fans, investors, and sponsors. Daddi et al. [33] further assert that coercive pressures often stem from stakeholders such as football institutions and governments, providing a basis for investigating stakeholder governance and its alignment with sustainability objectives in football organizations. Therefore, understanding the dynamics of stakeholder engagement and governance is crucial for fostering sustainable practices and effectively addressing the diverse interests and pressures within the football industry.

## 3 Methodology

Bibliometric research is a type of systematic literature review that utilizes quantitative and statistical methods to analyze bibliographic data. By employing quantitative measures, utilizing databases, and leveraging software powered by big data analytics and machine learning, bibliometric studies offer a more objective and comprehensive approach compared to other types of reviews [45]. Bibliometric research commonly employs two primary categories of analytical techniques: performance analysis and science mapping. Performance analysis is used to evaluate productivity and impact, providing insights into the performance of authors, institutions, or journals. On the other hand, science mapping is a relational technique that reveals knowledge clusters and connections within a field, allowing researchers to identify key topics, trends, and collaborations. These techniques enable a comprehensive understanding of the scholarly landscape and facilitate informed decision-making in research and academia [46].

Bibliometric research, particularly through science mapping, can help identify and uncover knowledge clusters, which are groups of related concepts or topics that are interconnected within a specific domain. Furthermore, science mapping can clarify nomological networks, which represent the causal relationships between variables or constructs in a particular area of study. Science mapping also enables the analysis of social patterns within a field, including collaborations, co-authorship networks, and other social processes that support knowledge development. Moreover, science mapping allows for tracking trends in a field and can help identify crucial knowledge gaps, highlighting areas that have received less attention or are underdeveloped. On the other hand, bibliometric findings can be utilized for five practical purposes: assessing and reporting the productivity and impact of research contributors, determining the reach for coverage claims, identifying social dominance or hidden biases to guide improvement efforts, detecting anomalies for further investigation, and evaluating relative performance for fair decision-making. However, it is important for bibliometric research to identify gaps, conflicting results, and areas that have been underexplored, as well as consider the implications of the research for theory development and practical applications [45].

To obtain the documents that form the foundation of any systematic review, it is necessary to specify the eligibility criteria for the included documents, which should align with the research objectives. Therefore, the search methods should be clearly defined to ensure reliable results, draw conclusions, and support decision-making [47,48]. This systematic review follows the four phases recommended by the PRISMA (Preferred Reporting Items for Systematic Reviews and Meta-Analyses for Scoping Reviews) guidelines: identification, screening, eligibility, and inclusion [49].

In the PRISMA identification phase, the Scopus and Web of Science (WoS) databases were utilized due to their worldwide recognition and relevance in indexing [50]. These databases were selected to search for documents related to the concepts of “Sustainability,” “Governance,” and “Stakeholders.” It is worth noting that the concept of sustainability is often linked to terms such as “Corporate Social Responsibility,” “Corporate Sustainability,” and “Business Sustainability,” which, although not entirely synonymous, share certain similarities. Likewise, the search equation is limited according to the purpose of the article, including concepts of soccer or football, and their relationships with the concept of governance and stakeholders because governance is a concept that involves stakeholders by understanding itself as a complex matrix of interactions and interrelationships between different actors and between different sets of ideas and practices [51]. In order to set the number of records identified through database searching, this study employed the following search equation in search fields of the article title, abstract and keywords: (“Sustaina*" OR “Corporat* social respons*" OR “corporate sustaina*" OR “business sustaina*") AND (((“Governance*") AND ((“Soccer” OR “Football"))) OR ((“Stakeholder*") AND (“Soccer” OR “Football"))). This search was conducted at the middle of June 2023, yielding 98 papers in Scopus and 87 papers in the Web of Science Core Collection.

The screening phase of the PRISMA model defines the number of records after removing duplicates. For this, one duplicate document was identified in Scopus and 51 duplicates in Scopus and WoS, obtaining 133 documents, of which 46 are exclusive in Scopus, 36 are exclusive in WoS, and 51 are present in both databases. The eligibility phase sets the number of full-text articles assessed for eligibility and the number of full-text articles excluded, with reasons. Thus, two articles belonging to Scopus and WoS, one article belonging to Scopus and one article belonging to WoS were eliminated and moved away from the scope of this study since they dealt with American Football and NFL. Likewise, two articles were excluded, one from Scopus and one that belongs exclusively to Scopus because they deal with topics outside the scope of research such as Hawaiian fishpond and neglected tropical disease programs. The inclusion phase of the PRISMA method sets the number of studies included in qualitative and quantitative synthesis, which in this case was 127 documents, of which 44 are exclusive to Scopus, 35 are exclusive to WoS, and 48 are present in both databases.

Once the documents for the bibliometric analysis have been obtained, the metrics to be used are defined. In this case, the metrics are based on the main techniques from the bibliometric analysis toolbox presented by Donthu et al. [46] and Mukherjee et al. [45], as shown in Table 1. Then, these results are analyzed using a performance analysis and science mapping through publication-related metrics, citation-and-publication-related metrics, co-authorship analysis, and co-word analysis to examine the evolution of research approaches around stakeholder governance and sustainability in football.

**Table 1:** Metrics for the bibliometric analysis.

Category	Analytical techniques	Metrics
Performance analysis	Publication-related metrics	• Total publications • Number of active years of publication • Productivity per active year of publication • Number of contributing authors • Sole-authored publications • Co-authored publications • Collaboration index • Collaboration coefficient
	Citation-and-publication-related metrics	• Total citations • Average citations • Number of cited publications • Proportion of cited publications • Citations per cited publication • Most influential publications • h-index
Science mapping	Co-authorship analysis	• Social interactions or relationships among authors • Authors and authors affiliation
	Co-word analysis	• Existing relationships among topics

## 4 Results

The results of the bibliographic analysis are presented below according to the categories of performance analysis and science mapping.

### 4.1 Performance analysis

For a comprehensive overview, Fig. 1 illustrates the annual distribution of documents retrieved from the Scopus and WoS databases, totaling 127 documents over a span of 16 active years of scientific production. Publications were registered between 2007 and mid-2023, except for the year 2008. Fig. 1 demonstrates a significant increase in studies and research on stakeholder governance and sustainability in football in recent years, particularly within the last three years, which accounted for 55 documents, representing 43.3% of the total publications on this topic in Scopus and WoS.

**Fig. 1:** Documents per year.

Since this study focuses on the evolution of governance and sustainability in football, the analysis of publications spans from 2007 to mid-2023. These dates correspond to the initial publications found in Scopus and WoS and the date of the literature search conducted. The comprehensive study of this scenario includes various elements, such as the number of publications and citations, contributions by country/territory, the distribution of citations across journals, subject areas, as well as the exploration of general and emerging concepts. These components align with the bibliometric and content analysis methodologies, as outlined by He et al. [52]. Similarly, Fig. 1 depicts the timeline of active publication years, ranging from 2007 to mid-2023, covering a span of 16 years. It is worth mentioning that there was a notable absence of publications in the year 2008. Nonetheless, the research topic has consistently garnered attention from researchers and a diverse range of publication sources throughout the analyzed period.

Regarding the number of published papers, Fig. 1 illustrates the following trends. From 2007 to 2015, a total of 27 articles were published, averaging three documents per year. These publications accounted for 21.3% of the articles on stakeholder governance and sustainability in football indexed in the Scopus and WoS databases. Moving on to the period between 2016 and 2020, 45 documents were identified, with an average of nine publications per year. These publications represented 35.4% of the total publications on the research topic, indicating a significant increase of 66.7% compared to the 2007–2015 period. Furthermore, between 2021 and mid-2023, a total of 55 documents were published, averaging 22 documents per year. This demonstrates a further increase of 22.7% compared to the previous period (2016–2020). These findings reveal an exponential growth in the number of publications per year in recent years, reflecting the considerable interest shown by the scientific and academic community in the subject of stakeholder governance and sustainability in football. This upward trend positions it as a prominent and noteworthy area for research agendas.

Table 2 reveals that most documents addressing stakeholder governance and sustainability in football are primarily associated with the subject areas of Business, Management & Accounting (30.8%) and Social Sciences (24.2%). This observation highlights a predominant focus on administrative and social applications of the research topic. Additionally, there is a notable prevalence of documents in English, which aligns with the predominant document type—scientific articles indexed in high-impact international journals. Throughout the analyzed period, 84.3% of the published documents are articles, 5.5% are book chapters, 3.9% are conference papers, 3.1% are reviews, 2.4% are books, and 0.8% consist of editorial material. Furthermore, the analysis indicates that 52.8% of the documents examined offer some form of open access (gold, green, bronze, hybrid), making them freely available to the public. On the other hand, 47.2% of the documents require a subscription or payment to access the full content, limiting public access. This distribution underscores the varying accessibility of the literature on stakeholder governance and sustainability in football, with a significant portion of the research being openly accessible to readers.

**Table 2:** Subject area in 2007 and mid-2023.

Subject Area	% Ind.	% Accum.
Business, Management & Accounting	31%	31%
Social Sciences	24%	55%
Economics, Econometrics and Finance Decision Sciences Others	9%	64%
Environmental Sciences	8%	71%
Medicine	5%	76%
Decision Sciences	5%	81%
Health Professions	5%	85%
Others	15%	100%

The analysis conducted in this study identifies 323 authors, of which 40 authors are identified as contributors to two documents, indicating a significant number of researchers who are committed and dedicated to exploring the topic of stakeholder governance and sustainability in football. Further analyzing the collaboration aspect, it is identified that out of the examined documents, 108 are multi-authored, accounting for 85% of the selected documents for this study, while 15% of the documents are sole-authored publications. Additionally, the total number of authors in these multi-authored documents amounts to 378, resulting in a collaboration index of 3.5. This indicates that, on average, multi-authored documents in this field are produced through collaboration among 3.5 authors. This demonstrates the relevance and range of the subject in the scientific community and the potential for obtaining multiple perspectives, approaches, and contributions related to the research topic.

Regarding citation analysis, it should be noted that out of the selected documents, 44 are exclusively indexed in Scopus, 35 are exclusively indexed in WoS, and 48 are indexed in both Scopus and WoS. Therefore, the citation measurement in Scopus is based on 92 documents, while the citation measurement in WoS is based on 83 documents. Considering that the documents indexed in Scopus have received a total of 970 citations and the documents indexed in WoS have received 1052 citations, we obtain an average of 10.5 citations per document in Scopus and 12.7 citations per document in WoS. For the calculation of citations per cited publication, only the 67 documents that received citations in Scopus and the 66 documents that received citations in WoS are considered. The average number of citations per cited document is 14.5 in Scopus and 15.9 in WoS. Furthermore, in total, 97 documents (76.4% of the total selected) received citations in either Scopus, WoS, or both databases.

Table 3 presents the most cited papers in Scopus and WoS based on the average number of citations per year. It identifies 15 papers that have received over 5 citations per year on average in either database. Among these papers, four are published by Routledge, with the paper by Jamali et al. [53] being the most cited per year, receiving an average citation rate of 16.5 and 7.7 in Scopus and WoS, respectively. Additionally, Table 3 highlights three highly cited articles published in *European Sport Management Quarterly* (Routledge) [[54], [55], [56]], and two highly cited articles published in the *Journal of Sport Management* (Human Kinetics Publishers Inc.) [57,58]. Therefore, these journals can be considered high impact within the analyzed period.

**Table 3:** Most cited documents in Scopus and WoS.

Authors	Title	Source	Year	Cites		Average cites per year	
				Scopus	WoS	Scopus	WoS
[53]	CSR Institutionalized Myths in Developing Countries: An Imminent Threat of Selective Decoupling	Business and Society (Sage)	2017	107	50	16.5	7.7
[58]	Corporate Social Responsibility in Professional Team Sports Organizations: An Integrative Review	Journal of Sport Management (Human Kinetics Publ)	2018	–	59	–	10.7
[59]	Clusters, Chains and Compliance: Corporate Social Responsibility and Governance in Football Manufacturing in South Asia	Journal of Business Ethics (Springer)	2010	124	117	9.2	8.7
[60]	Knowledge management and intellectual capital in knowledge-based organizations: a review and theoretical perspectives	Journal of Knowledge Management (Emerald)	2020	–	26	–	7.4
[54]	Organizational learning for corporate social responsibility in sport organizations	European Sport Management Quarterly (Taylor & Francis)	2019	–	31	–	6.9
[55]	The impact of UEFA financial fair play on player expenditures, sporting success and financial performance: evidence from the Italian top league	European Sport Management Quarterly (Routledge)	2021	16	–	6.4	–
[61]	Labor agency in the football manufacturing industry of Sialkot, Pakistan	Geoforum (Pergamon-Elsevier)	2013	–	64	–	6.1
[3]	Stimulating the adoption of green practices by professional football organizations: a focus on stakeholders' pressures and expected benefits	Sport Management Review (Taylor & Francis)	2023	2	3	4.0	6.0
[56]	Management strategies of non-profit community sport facilities in an era of austerity	European Sport Management Quarterly (Taylor & Francis)	2019	–	26	–	5.8
[62]	The profitable relationship among corporate social responsibility and human resource management: A new sustainable key factor	Corporate Social Responsibility and Environmental Management (Wiley)	2020	19	18	5.4	5.1
[63]	Assessing the role and use of recycled aggregates in the sustainable management of construction and demolition waste via a mini-review and a case study	Waste Management and Research (Sage)	2020	19	18	5.4	5.1
[64]	Labour in Global Value Chains: Work Conditions in Football Manufacturing in China, India and Pakistan	Development and Change (Wiley)	2012	–	62	–	5.4
[65]	Sport for development and peace as contested terrain: place, community, ownership	International Journal of Sport Policy and Politics (Routledge)	2014	51	–	5.4	–
[57]	Applying a communicating vessels framework to csr value co-creation: Empirical evidence from professional team sport organizations	Journal of Sport Management (Human Kinetics Publishers Inc.)	2016	35	40	4.7	5.3
[66]	A combined methodology for the concurrent evaluation of the business, financial and sports performance of football clubs: the case of France	Annals of Operations Research (Springer)	2018	29	24	5.3	4.4

Lund-Thomsen is the author with the highest impact, contributing the highest number of the most cited documents [53,59,61,64], and receiving a total of 231 citations in Scopus and 293 citations in WoS. Anagnostopoulos also contributes three of the most cited documents [54,57,58], accumulating a total of 35 citations in Scopus and 130 citations in WoS. Therefore, it can be concluded that these authors are the most influential and impactful contributors in the field of stakeholder governance and sustainability in football. Table 3 also reveals the contribution of authors such as Nadvi, who is a co-author with Lund-Thomsen, and Khara, who is a co-author with Lund-Thomsen in two of the most cited documents [53,59,64,64] respectively. This indicates their significant involvement and impact in the field of stakeholder governance and sustainability in football.

The literature on stakeholder governance and sustainability in football has been published in 86 sources, highlighting *European Sport Management Quarterly* and *Sustainability (Switzerland)* in Table 4, with nine papers each. They are followed by *Frontiers in Sports and Active Living* and *Soccer and Society*, each with five papers. Additionally, the *Journal of Business Ethics* has four papers on the topic. Table 4 further reveals that *Routledge* is the publisher contributing to three out of the 15 leading journals, while *MDPI*, *Springer*, *Emerald*, and *Taylor and Francis* contribute to two leading journals each.

**Table 4:** Leading journals and publishers.

Source Title	Publisher	Docs.
European Sport Management Quarterly	Routledge	9
Sustainability (Switzerland)	MDPI	9
Frontiers in Sports and Active Living	Frontiers Media	5
Soccer and Society	Routledge	5
Journal of Business Ethics	Springer	4
Corporate Social Responsibility and Environmental Management	John Wiley and Sons	3
Journal of Sport Management	Human Kinetics Publ Inc	3
Sport Management Review	Elsevier	3
Sport, Business and Management: An International Journal	Emerald	3
CSR, Sustainability, Ethics and Governance	Springer	2
International Journal of Financial Studies	MDPI	2
International Journal of Sport Policy and Politics	Taylor and Francis	2
International Journal of Sports Marketing and Sponsorship	Emerald	2
Journal of Sport and Tourism	Roultedge	2
Managing Sport and Leisure	Taylor and Francis	2

Table 5 presents the most cited journals in this research, with *European Sport Management Quarterly* (Routledge) standing out once again, contributing three of the most cited papers and having an h-index of 6. This indicates that at least 6 of the papers published in this journal have received 6 or more citations. Other notable journals include *Journal of Business Ethics* (Springer), which provides one of the most cited papers in Table 3 [59] and has an h-index of 3, *Business and Society* (Sage), which provides the article with the highest average citations per year [53], and *Journal of Sport Management* (Human Kinetics Publ), which provides two of the most cited papers. These journals are recognized for receiving over 100 citations in Scopus and/or WoS. Therefore, the journals listed in Table 5 are important sources for publishing research on stakeholder governance and sustainability in football due to their visibility and high citation impact.

**Table 5:** Most cited journals.

Journal	Cites Scopus	Cites Wos	h-index
European Sport Management Quarterly (Taylor & Francis)	108	191	6
Journal of Business Ethics (Springer)	154	171	3
Business and Society (Sage)	107	50	1
Journal of Sport Management (Human Kinetics Publ)	35	102	3
Geoforum (Pergamon-Elsevier)	–	64	1
Development and Change (Wiley)	–	62	1
Sustainability (MDPI)	49	61	5
International Journal of Sport Policy and Politics (Routledge)	59		2
Journal of Management and Organization (Cambridge Univ Press)	54	55	1
Corporate Social Responsibility and Environmental Management (Wiley)	42	36	2

### 4.2 Science mapping

Table 6 shows that Lund-Thomsen and Anagnostopoulos stand out as leading authors with six documents each. Both authors not only emerge as the leading authors in the research topic but also contribute the highest number of most cited documents, as indicated in Table 3. They are followed by Willem with five documents, and Constandt and Kolyperas with four documents each. Additionally, several authors are noted for their contribution of three documents each, including Daddi, Gray, Morrow, Samuel, Sparks, Thomas, Todaro, and White.

**Table 6:** Leading contributing authors.

Authors	Affiliation	Country	Databases			Total Docs.
			Scopus	WoS	Scopus and WoS	
Anagnostopoulos, C.	Molde University College	Norway	–	[54,58,67,68]	[57,69]	6
Lund-Thomsen, P.	Copenhagen Business School	Denmark	[70]	[61,64,71]	[53,59]	6
Willem, A.	Ghent University	Belgium	–	[54,[72], [73], [74]]	[75]	5
Constandt, B.	Ghent University	Belgium	–	[[72], [73], [74]]	[75]	4
Kolyperas, D.	University of Stirling	United Kingdom	[76,77]	[67]	[57]	4
Daddi T.	Sant’Anna School of Advanced Studies	Italy	–	–	[3,10,33]	3
Morrow S.	University of Stirling	United Kingdom	[77]	[14]	[78]	3
Samuel A.	Cardiff University	United Kingdom	–	[79]	[80,81]	3
Sparks L.	University of Stirling	United Kingdom	[76,77]	–	[57]	3
Thomas R.J.	Aston University	United Kingdom	–	[79]	[80,81]	3
Todaro N.M.	Sant’Anna School of Advanced Studies, Pisa, Italy	Italy	–	–	[3,10,33]	3
White G.R.T.	Cranfield University	United Kingdom	–	[79]	[80,81]	3

Among the documents published from 2007 to mid-2023, the Molde University College and Copenhagen Business School emerge as the leading affiliations, with each institution being associated with six documents from the leading authors. Ghent University follows closely with its presence in five documents. The University of Sterling is credited in four papers from the leading authors, while Cardiff University and Sant’Anna School of Advanced Studies contribute to three documents each. Table 7 provides additional insights into the institutions that have made significant contributions to the research topic. The University of Stirling, based in Scotland, takes the lead with a participation rate of 5.5% in the publications [14,57,76,78,[82], [83], [84]], including contributions from leading authors like Kolyperas and Sparks. Coventry University [56,60,69,85], Texas A&M University [3,[86], [87], [88]], and the University of Manchester [59,64,69,89] also emerge prominently, each with four publications to their credit. It is worth noting that the leading authors and their affiliations are primarily concentrated in Europe, specifically in countries and territories such as the United Kingdom, Norway, Denmark, Belgium, Italy, Germany, and Cyprus. Among the leading affiliations, one institution from the United States stands out. These institutions demonstrate their active involvement and expertise in the field of stakeholder governance and sustainability in football, contributing to the body of knowledge through their research outputs.

**Table 7:** Leading affiliations.

Affiliation	Docs	% Docs^a^
University of Stirling (United Kingdom)	7	5.5%
Copenhagen Business School (Denmark)	6	4.7%
Molde University College (Norway)	6	4.7%
Ghent University (Belgium)	5	3.9%
Coventry University (United Kingdom)	4	3.1%
Texas A&M University (USA)	4	3.1%
University of Manchester (United Kingdom)	4	3.1%
Aston University (United Kingdom)	3	2.4%
Cardiff University (United Kingdom)	3	2.4%
German Sport University Cologne (Germany)	3	2.4%
Sant’Anna School of Advanced Studies (Italy)	3	2.4%
University of Glasgow (United Kingdom)	3	2.4%
University of Liverpool (United Kingdom)	3	2.4%
University of London (United Kingdom)	3	2.4%
University of Nicosia (Cyprus)	3	2.4%

a *Documents in which one or several authors with corresponding institutional affiliation participate.*

Among the funding organizations supporting studies on stakeholder governance and sustainability in football, the European Commission (EC) emerges as a notable contributor, backing three papers [3,10,33] authored by Daddi, Rizzi, Pretner, Todaro, Annunziata, Frey, and Iraldo, who are affiliated with institutions such as Sant'Anna School of Advanced Studies (Italy), Texas A&M University (USA), and the University of Perugia (Italy). Additionally, there are 20 other funding organizations identified as sponsors of studies related to the research topic. These funding organizations play a crucial role in advancing research and promoting understanding in the field of stakeholder governance and sustainability in football.

Collaborative networks can be observed within the field of stakeholder governance and sustainability in football. Anagnostopoulos and Kolyperas have collaborated on issues related to CSR value co-creation from a consumer culture theory perspective, as well as strategic decision-making in charitable foundations in English football [57,67]. Lund-Thomsen and Nadvi have worked together on various topics such as corporate social responsibility (CSR), global value chains, industrial clusters, production networks, governance, trade, and globalization [59,64]. Willem and Constandt, both from Ghent University (Belgium), have co-authored studies on the longitudinal analysis of code effectiveness in football clubs to counteract unethical behavior and the role of ethical leadership among football club fans [72,73]. They have also explored network structures and governance through cause-related marketing in professional football teams, examining CSR management from an entrepreneurship perspective [74,75].

Kolyperas, Sparks, and Morrow have collaborated on research related to corporate governance, CSR, stakeholders, and organizational change [77]. Kolyperas and Sparks have also worked together on studies focusing on CSR communication, sport management, sports marketing, and corporate governance [57,76]. Daddi and Todaro from Sant'Anna School of Advanced Studies (Italy) have conducted research on the relationship between sport and sustainability, specifically examining the reduction of environmental impact in sports events and the influence of institutional pressures on the adoption of environmental practices by football organizations [10,33]. They have also investigated the drivers and expected outcomes of environmental practices adopted by football organizations [3]. Thomas, Samuel, and White, from the United Kingdom, have collaborated on various topics, including football places, football as a catalyst for change, and the incorporation of sustainability in mainstream business and marketing education [80,81]. They have also co-authored a study on the concept of supererogation as a means to address social and environmental goals beyond CSR [79].

When examining the most frequent keywords, Fig. 2 illustrates that the most used concept is CSR, appearing in 44 documents. It is closely followed by football, which is mentioned in 27 documents. Sustainability and financial management are each present in 12 documents. Additionally, the concepts of football clubs, stakeholder theory, and stakeholders are found in 10 or more documents, indicating their significance in the research topic. Other keywords such as community, social impact, social responsibility, ethics, professional football, and football industry also feature prominently, appearing in five or more documents, emphasizing their relevance to the central theme.

**Fig. 2:** Most recurrent keywords for stakeholder governance and sustainability in football.

The bibliographic coupling allows the identification of the main topics and research concepts from 2007 to 2023 through a co-occurrence analysis for keywords and co-authorships based on clusters generated with the VOSviewer software, identifying research nodes in each cluster through the size of its corresponding spheres. Fig. 3 depicts the co-occurrence analysis of the main concepts related to stakeholder governance and sustainability in football from 2007 to mid-2023. The analysis reveals five distinct clusters: governance, CSR, organization, football, and sport. The input database for the analysis was compiled by gathering keywords from Scopus and WoS documents and consolidating similar concepts. For example, concepts such as corporate social responsibility, corporate social-responsibility, CSR, and social responsibility were unified under the term CSR. Similarly, terms like stakeholder, stakeholders, and stakeholder theory were grouped under the category of stakeholders. Additionally, the terms football and soccer were combined as football, and sport and sports were unified as sport. Lastly, football clubs and clubs were considered as football clubs.

**Fig. 3:** Co-occurrence analysis of concepts and keywords.

The Vosviewer software was configured to conduct a co-occurrence analysis using the following parameters: type of analysis - co-occurrence, counting method - full counting, and unit of analysis - all keywords. The analysis was conducted on a total of 127 documents, resulting in a collection of 747 keywords. Out of these, 22 keywords met the predefined threshold of a minimum of five occurrences. Table 8 presents the data on total link strength and occurrence between keywords, which enabled the identification of five clusters. The clusters were named based on the core keyword with the highest total link strength and occurrence within each cluster.

**Table 8:** Findings of the co-ocurrence analysis.

Cluster	Keywords of the clusters	Occurrences	Total links strength
***Cluster 1***	Governance	21	74
	Performance	10	42
	Sport organizations	7	24
	Business	5	23
	Efficiency	5	19
	Financial fair play	5	16
***Cluster 2***	CSR	53	129
	Football	38	93
	Stakeholder	23	59
	Ethics	6	19
	Stakeholder management	5	14
***Cluster 3***	Organization	7	38
	Determinants	6	34
	Professional sport	8	28
	Sport management	5	12
***Cluster 4***	Football clubs	17	58
	Management	7	35
	Theory	6	33
	Community	6	21
***Cluster 5***	Sport	19	50
	Sustainability	16	48
	Sustainable development	7	7

*Items of keywords – 22; Number of clusters – 5; Total links strength - 876*.

The Governance cluster (red) presented in Fig. 4(a) indicates that the governance concept meets with concepts like performance, financial fair play, efficiency, sports organizations, and business. The CSR cluster (green) involves the keywords with the highest link strength, which indicates the number of publications in which two keywords occur together. Fig. 4(b) indicates that the keyword CSR meets in the analyzed documents with concepts like football, stakeholders, ethics, and stakeholder management. The Organization cluster (blue) shown in Fig. 4(c) meets the concept of organizations with concepts such as determinants, professional sport, and sport management. The Football clubs cluster (yellow) shown in Fig. 4(d) has the concept of football clubs as its central node and is directly related to management, theory, and community. The Sport cluster (purple) shown in Fig. 4(e) has the concept of sport as its central node and is directly related to sustainability and sustainable development.

**Fig. 4:** (a) Cluster 1 red; (b) cluster 2 green; (c) cluster 3 blue; (d) cluster 4 yellow; (e) cluster 5 purple.

## 5 Discussions

Through a comprehensive bibliometric analysis, the importance and significance of stakeholder governance and sustainability in football have been highlighted. The utilization of renowned databases such as Scopus and WoS has provided access to valuable and impactful literature, making them crucial for conducting rigorous systematic literature reviews and bibliometric analysis in this research field [50,52]. Moreover, the increasing number of publications found in both databases reflects the growing academic and scientific interest in the topic. This indicates that there is still ample room for further exploration and examination of various aspects related to stakeholders, governance, and sustainability in football. Regarding the lead authors, Lund-Thomsen and Anagnostopoulos have emerged as highly influential and prominent authors in the field of stakeholder governance and sustainability in football. They not only contribute a significant number of the most cited documents but also play a central role in shaping research in this area. It is also worth noting that Nadvi and Khara have made notable contributions as co-authors with Lund-Thomsen, further enriching the literature on the subject.

During the analyzed period, it is observed that collaboration among authors is prevalent, with an average of 3.5 authors per document. Networks have been identified among prominent authors across various topics such as CSR, corporate governance, stakeholders, global value chains, production networks, trade and globalization, organizational change, sport management, marketing, value co-creation of professional football clubs, consumer culture theory, charitable foundations in English football, code effectiveness in football clubs, ethical leadership of football club supporters, public relations, media presence, relationship between sport and sustainability, environmental impact reduction in football events, drivers and expected outcomes of environmental practices adopted by football organizations, football as a catalyst for change, and supererogation events. These collaborations and networks contribute to the interdisciplinary nature of research in this field and promote knowledge exchange and advancement.

The leading affiliations of the published papers in the research topic are primarily concentrated in Europe, particularly in the United Kingdom. Prominent institutions include the University of Stirling, Coventry University, University of Manchester, Aston University, Cardiff University, University of Glasgow, University of Liverpool, and University of London. Other European institutions contributing significantly to the research topic are Copenhagen Business School in Denmark, Molde University College in Norway, Ghent University in Belgium, Sant’ Anna School of Advanced Studies in Italy, German Sport University Cologne in Germany, and the University of Nicosia in Cyprus. Notably, Texas A&M University from the United States also stands out as a leading affiliation outside of Europe. These institutions demonstrate their active engagement in researching stakeholder governance and sustainability in football, contributing to the advancement of knowledge in the field.

The bibliometric analysis reveals that *European Sport Management Quarterly* is the most prominent journal in the field of stakeholder governance and sustainability in football. Not only does it publish a substantial number of research articles on the topic, but it also features highly cited articles, earning it an h-index of 6. Other notable journals include *Journal of Business Ethics* with an h-index of 3, *Journal of Sport Management* (which contributes two of the most cited papers), *Business and Society* which provides the article with the highest average citations per year, as well as *Sustainability (Switzerland)*, *Frontiers in Sports and Active Living*, and *Soccer and Society*, which contribute a significant number of articles to the research field. Routledge emerges as the most influential publisher during the analyzed period, publishing not only the journals with the highest number of documents but also some of the most cited articles. Additionally, the European Commission stands out as the primary sponsor of studies on stakeholder governance and sustainability in football, providing support for three documents. The subject areas in which most of the documents are categorized include Business, Management & Accounting, and Social Sciences.

The keyword analysis revealed that the most addressed concepts in the research documents are CSR, football, sustainability, financial management, football clubs, stakeholder theory, and stakeholders. The co-occurrence analysis further identified five clusters that represent the main concepts within the research topic: governance, CSR, organization, football, and sport. These clusters demonstrate the interrelationships between different concepts. Governance is associated with performance, efficiency, business, and sport organization. CSR is frequently linked to themes of stakeholders and ethics. The concept of organizations is connected to determinants, professional sport, and sport management. Football clubs are often discussed in relation to management, theory, and community. Finally, the sport cluster encompasses themes of sustainability and sustainable development. These findings provide insights into the key concepts and their interconnections within the field of stakeholder governance and sustainability in football.

The concepts of CSR and sustainability are being approached as distinct topics [37], with corporate sustainability being seen as an evolution of CSR. Corporate sustainability goes beyond the philanthropic nature of CSR by encompassing the needs of future generations. This aligns with the definition of sustainable development in the Bruntland declaration, which emphasizes meeting present needs without compromising the ability of future generations to meet their own needs. The issues related to sustainability are typically presented through the interaction of various dimensions, including economic, social, environmental, and institutional aspects [90]. In the context of corporate sustainability, it encompasses both present and future performance of the company [91]. In the short term, it involves minimizing economic, social, and environmental impacts, while in the long term, it involves governance that considers the ethical and political stance of the company [41]. In the context of football, this means that football club managers may incorporate sustainability into their business models in response to stakeholder pressure, as stakeholders have a significant influence on the expected sustainability outcomes [4,33]. This framework provides a basis for research on stakeholder pressure in national football teams and football clubs across different contexts and regions globally, highlighting the importance of understanding the influence of stakeholders and their role in shaping sustainability efforts in football.

Regarding literature reviews that connect CSR with football, notable works include Dimitropoulos and Vrondou [92], Fifka and Jaeger [93], and Walzel et al. [58]. Dimitropoulos and Vrondou [92] emphasize four key dimensions of CSR that sports companies should prioritize to enhance their reputation: community engagement, environmental protection, product and service quality, and stakeholder satisfaction and retention. Similarly, Fifka and Jaeger [93] identify six areas of CSR that have been explored in the football industry: community involvement, human capital, fan and member relations, business environment, compliance, and ecological environment. Additionally, Walzel et al. [58] highlight that CSR in sports research has predominantly focused on social programs and community relations. It is worth noting that the first two studies connect CSR with the environment, indicating overlapping topics between CSR and sustainability. On the other hand, literature reviews that explore the association between sustainability and football, noteworthy works include the review by Mabon [94] where an extensive analysis identifies four research areas: the impact of football on climate, the impact of weather on football, football as a driver of pro-environmental actions, and the relationship between football and carbon-intensive sports. Another review by Annesi et al. [95] reveals that sport's contribution to the 2030 Agenda is strategically significant; however, there is a lack of consideration for SDGs in the sports literature.

The focus on sustainability in football has traditionally been centered on financial sustainability, given the significant financial implications within the industry, including high player salaries and the impact of the Covid-19 pandemic on club finances [96,97]. However, in recent years, there has been a notable shift towards studying environmental sustainability in football, particularly in the period from 2021 to mid-2023. Researchers have applied the “Pressure Framework” to understand the motivations behind sports organizations, including football clubs, striving to achieve sustainability objectives, particularly in the environmental domain. These studies emphasize the importance of managing the pressures exerted by various stakeholders, highlighting the necessity of stakeholder governance to fulfill sustainability goals. Notably, the works of de Fernández-Villarino [5], Daddi et al. [33], Daddi et al. [10], McCullough and Cunningham [4], and Cayolla et al. [21] have made significant contributions to advancing the conceptualization and measurement of the effects of stakeholder pressures on environmental sustainability. Some of these studies even argue for the potential of football to act as agents of social change by fostering environmental awareness, transcending behaviors within stadiums and influencing the personal lives of fans [30].

It is indeed noteworthy that the number of bibliometric studies specifically addressing the integration of sustainability and governance of stakeholders in football is limited. One of the few existing studies is conducted by Escamilla-Fajardo et al. [98], where four main areas of research are identified in the field of football sustainability: football, entrepreneurship, and social development; football, innovation, and management; football, efficiency, and new technologies; and football, injuries, and innovation in rehabilitation. Similarly, Gónzalez-Serano et al. [99] identified seven central themes, with sports mega-events and sustainability being the sub-area that has received the most attention in terms of research, followed by sports innovation for inclusion. Although these literature reviews and bibliometric analyses provide valuable insights, they do not comprehensively address the intertwined issues of sustainability and governance stakeholders in football. Therefore, this review aims to contribute to the development of this specific field of study by offering a comprehensive examination of the topic.

### 5.1 Future research lines and limitations of the study

Upon reviewing several of the documents analyzed in this bibliometric analysis, it is evident that the relationship between sustainability and football predominantly focuses on financial sustainability and environmental sustainability. This observation highlights the ample research opportunities in social sustainability, aligning with the recommendations of Trendafilova and McCullough [100]. Therefore, future research is encouraged to explore the dimensions of economic, social, and environmental sustainability using the triple bottom approach. Furthermore, it is proposed that future studies generate theoretical and methodological frameworks that address the co-creation of value [34] or joint creation of value [101] within the context of football. These frameworks should acknowledge the significance of stakeholder governance in facilitating value co-creation, providing insights into how different stakeholders can collaborate and contribute to sustainable outcomes.

Another proposed research line is to investigate the effects of pro-environmental regulations on the adoption of sustainability policies in the football sector, which aligns with Jager's recommendations [39]. Initial explorations in this field have been presented in the works of Daddi et al. [33] and Daddi et al. [10], revealing a positive relationship between governance practices and coercive pressures. These coercive pressures may be linked to regulations established by football and government institutions. It is important to acknowledge that McCullough and Cunningham (4) mentioned that the pressures exerted can be of mimetic nature (imitation), coercive nature (resulting from compliance with regulations), and normative nature (related to what is deemed appropriate). Therefore, it is suggested that future studies not only focus on normative pressures stemming from regulations but also explore mimetic and normative pressures in the context of sustainability and governance in football.

Additionally, future research includes studying specific stakeholders, particularly fans, who, due to their emotional connection with football teams or clubs, could play a crucial role in achieving sustainability objectives within stadiums. Research can focus on exploring initiatives aimed at waste reduction and promoting recycling [101]. It is also suggested to conduct case studies or quantitative studies to evaluate the impact of these environmental initiatives on the development of environmental awareness among fans. Understanding the relationship between environmental initiatives and fan behavior can serve as a catalyst for social change [30].

Likewise, future research is proposed to identify barriers to the governance of stakeholders in the football sector. While some studies have linked governance failures in football to issues such as communication and lack of participation, primarily from fans [26,102], there is still significant potential to expand this line of inquiry to other stakeholders. This includes investigating the role of investors, local communities, governments at various levels, and football institutions in the governance process. Furthermore, there is a need for studies that evaluate the types of governance practices adopted by management teams of football teams or clubs, as well as the broader institutions within the football sector.

On the other hand, this study acknowledges certain limitations. Firstly, the bibliometric analysis relied on the selected databases, Scopus and WoS, which may have excluded relevant publications from other sources. Secondly, the analysis focused on specific keywords and criteria, which might have overlooked certain aspects of stakeholder governance and sustainability in football. This observation raises the concern that the results primarily represent European football, potentially indicating a lack of studies on sustainability and governance of stakeholders in football leagues in Central and South America, as well as in Asia and Africa. It is essential to address this research gap and expand the scope of future studies to encompass these regions and gain valuable insights into the specific challenges, opportunities, and practices in these contexts. This will contribute to a more comprehensive understanding of the global landscape of sustainability in football and provide valuable knowledge for decision-makers, stakeholders, and policymakers in these regions.

### 5.2 Implications for the application of environmental and sustainability policies in football

The governance of stakeholders has the potential to be an effective tool for implementing pro-environmental actions and generating positive impacts in the football industry. These actions can be carried out within the context of football stadiums or in broader sporting events, and they have the potential to influence the personal lives of individuals within the various stakeholders involved. Fans can play a crucial role in promoting environmental awareness and sustainable behaviors due to their emotional connection with their teams. Engaging fans and other stakeholders in sustainability initiatives requires collaborative efforts and effective management of their sentiments and interests. By fostering a sense of shared responsibility and creating platforms for participation, football organizations can harness the passion and loyalty of fans to drive positive environmental change. Furthermore, involving other stakeholders such as investors, local communities, and football institutions in collaborative efforts can enhance the effectiveness and impact of sustainability initiatives.

Because football industry companies operate within a legal and regulatory framework, both governments and football institutions are required to develop proactive regulations that encourage these companies to adopt pro-environmental practices or more broadly, promote compliance with the SDGs. In the context of football, these regulations can align with SDG 12 (Responsible Consumption and Production), SDG 13 (Climate Action), as well as address effects related to social and economic dimensions. For instance, initiatives aimed at eliminating racism in football or empowering women's football can contribute to the achievement of SDG 10 (Reduced Inequalities) and SDG 5 (Gender Equality) respectively.

It is crucial for governments and football institutions to collaborate in creating regulatory frameworks that incentivize football companies to integrate sustainability practices into their operations and decision-making processes. Consequently, the industry can contribute to the global sustainability agenda, and these regulations can foster responsible and ethical behavior, promote social inclusivity, and ensure that the football industry plays a positive role in broader societal goals.

## 6 Conclusions

This study presented a bibliometric analysis on stakeholder governance and sustainability in football using two of the most relevant and widely accepted databases in the scientific community: Scopus and WoS. The bibliometric analysis yielded 127 documents for analysis, 44 of them in Scopus, 35 in WoS, and 48 in Scopus and WoS to determine the publication-related metrics, citation-related metrics, and bibliographic coupling. The findings indicate that Lund-Thomsen and Anagnostopoulos stand out as the leading authors with the most published papers and most cited papers related to stakeholder governance and sustainability in football. The collaboration among authors in this topic is prevalent with an average of 3.5 authors per document, addressing topics such as CSR, corporate governance, stakeholders, global value chains, production networks, trade and globalization, organizational change, sport management and marketing, value co-creation of professional football clubs, consumer culture theory, ethical leadership of football club supporters, public relations, media presence, environmental impact reduction in football events, football as a catalyst for change, among others. In addition, Business, Management & Accounting, and Social Sciences stand out as the thematic areas where most research on stakeholder governance and sustainability in football is conducted.

This study also identified that the institutions with the most research on stakeholder governance and sustainability in football are in European countries, in the United Kingdom. Researchers interested in the subject of this research can consult journals such as *European Sport Management Quarterly*; *Journal of Business Ethics; Journal of Sport Management; and Business and Society* which provides the article with the highest average citations per year. Regarding the keywords and main concepts, the bibliometric analysis showed that the research topics mainly revolve around CSR, football, sustainability, financial management, football clubs, stakeholder theory, and stakeholders. Likewise, the concepts and keywords were grouped into clusters of governance, CSR, organization, football, and sport. The results reveal a scarcity of comprehensive documents that address the intertwined issues of sustainability and stakeholder governance in football. Instead, the existing literature tends to separately address reviews of CSR and football, sustainability and football, or governance and football. Therefore, there is a gap in the literature that calls for more comprehensive studies that integrate the concepts of sustainability and stakeholder governance within the context of football.

Future research is encouraged to explore the dimensions of economic, social, and environmental sustainability using the triple bottom approach and to acknowledge the significance of stakeholder governance in facilitating value co-creation. This will provide insights into how different stakeholders can collaborate and contribute to sustainable outcomes. Likewise, future studies should identify barriers to stakeholder governance in the football sector, going beyond normative pressures stemming from regulations, and explore mimetic and normative pressures in the context of sustainability and governance in football. Finally, involving other stakeholders such as investors, local communities, and football institutions in collaborative efforts can enhance the effectiveness and impact of sustainability initiatives. Consequently, the football industry can contribute to the global sustainability agenda by fostering responsible and ethical behavior, promoting social inclusivity, and ensuring that the football industry plays a positive role in broader societal goals.

## Author contribution statement

All authors listed have significantly contributed to the development and the writing of this article.

## Data availability statement

Data will be made available on request.

## Additional information

No additional information is available for this paper.

## Declaration of competing interest

The authors declare that they have no known competing financial interests or personal relationships that could have appeared to influence the work reported in this paper.
